# *Dysosma versipellis* Extract Inhibits Esophageal Cancer Progression through the Wnt Signaling Pathway

This article has been retracted.

**DOI:** 10.1155/2021/1221899

**Published:** 2021-10-20

**Authors:** Yanchun Pu, Ping Jin, Lianghong Liu, Qinlin Pu, Fangping Wu

**Affiliations:** School of Pharmaceutical Sciences, Hunan University of Medicine, No. 492, Jinxi South Road, Huaihua, Hunan Province 418099, China

## Abstract

**Objective:**

In this study, we aim to investigate the effect of *Dysosma versipellis* extract on biological behavior of esophageal cancer cells and its underlying mechanisms.

**Methods:**

A total of 30 BALB/C nude mice (class SPF) were equally and randomly divided into the control group, model group, and *Dysosma versipellis* group. CP-C cell of esophageal cancer was subcutaneously injected into the model group as well as the *Dysosma versipellis* group, and the same amount of normal saline into the control group, in order to compare the tumorigenesis of nude mice of three groups. Wnt, *β*-catenin, and p-GSK3*β*/GSK3*β* expression in tumor tissues was detected using Western blot. CP-C cells in logarithmic growth were selected and divided into 4 groups, including the control group, podophyllotoxin group, Wnt activator group, and combined group (mixture of podophyllotoxin and Wnt activator). The cell viability, apoptosis, and invasion ability, Wnt, *β*-catenin, and p-GSK3*β*/GSK3*β* expression level of CP-C cells in each group were detected via MTT assay, flow cytometry, transwell, and Western blot, respectively.

**Results:**

The tumorigenesis rates of the control group, model group, and *Dysosma versipellis* group were 0%, 90% (1 tumor-free mouse), and 80% (2 tumor-free mice), respectively. The tumor mass in the *Dysosma versipellis* group was significant less than that in the model group. Based on the results of Western blot, Wnt, *ß*-catenin, and p-GSK3*β*/GSK3*β* expression of the *Dysosma versipellis* group was lower than that of the control group. The in vitro viability test indicated that there was a significant difference in cell viability exhibited among four groups. Cell viability level in the 3 groups, including the combined group, blank group, and Wnt activator group, was higher than the podophyllotoxin group at each time point. In vitro apoptosis assay revealed that significant differences in cell apoptosis exhibited among four groups. Cell apoptosis rate was higher in the podophyllotoxin group compared to the remaining three groups. The Wnt activator group showed the lowest cell apoptosis rate. The in vitro invasion assay demonstrated that numbers of transmembrane cell in the 3 groups, involving the combined group, blank group, and Wnt activator group, showed a higher level than the podophyllotoxin group. The results of Western blot manifested that the podophyllotoxin group showed lower level of Wnt, *ß*-catenin, and p-GSK3*β*/GSK3*β* expression compared to the other 3 groups.

**Conclusion:**

Podophyllotoxin in *Dysosma versipellis* has an excellent antiesophageal cancer effect and is able to inhibit cell viability as well as invasion ability and promote apoptosis of esophageal cancer cells by inhibiting the Wnt signaling pathway, which could be potentially used in future clinical treatment of esophageal cancer.

## 1. Introduction

Esophageal cancer is one of the most common epithelial malignancies in the digestive system, mainly composed of squamous cell carcinoma and adenocarcinoma, which affects more than 450,000 people worldwide [1]. It ranks the eighth among most common cancers and sixth among life-threatening cancers [2]. Despite the progresses have been made in radiotherapy, chemotherapy, neoadjuvant therapy, and immunotherapy, the patients with esophageal cancer have poor prognosis, with 15–25% overall 5-year survival [3]. The esophageal cancer patients with poor prognosis are associated with advanced diagnosis and metastatic tendency, even if the tumor is superficial [4]. In recent years, many scholars have determined the therapeutic effect of Chinese herbal extracts on tumors, with less toxicity and side effects [5, 6], in which *Dysosma versipellis* has gained great popularity as an antitumor drug. Khaled et al. [7] have documented that *Dysosma versipellis* extract, deoxypodophyllotoxin, can inhibit proliferation of breast cancer cells by interfering with the cell cycle to regulate proteins such as cyclin B1, CDC25c, and CDK1, as well as destroying cytoskeleton and inducing cell cycle arrest in G2/M. This regulatory mechanism is similar to the results reported by Juan et al. [8], that is, in G2/M, podophyllotoxone extracted from *Dysosma versipellis* inhibits the proliferation of prostate cancer cells by blocking cell cycle. Podophyllotoxin, as another extract of *Dysosma versipellis*, shows significant excellent activity to drug-sensitive and drug-resistant or even multidrug-resistant cancer cells by inhibiting tubulin polymerization. Podophyllotoxin and its derivatives are mainly used as strong antiviral drugs and antitumor drugs [9, 10]. However, few reports have been done on the effect of podophyllotoxin in esophageal cancer, and its specific role in esophageal cancer remains unclear. Wnt signaling represents one of a series of pathways, including notch Delta, hedgehog, transforming growth factor B/bone morphogenetic protein, and hippo. Wnt signaling has become a basic growth control pathway in various fields from cancer and development to early animal evolution [11]. It is associated with inducing cell proliferation and forming growth tissue, which plays a role as a directional growth factor in this process [10, 12, 13]. Reportedly, inhibiting typical Wnt signaling pathways could promote apoptosis in esophageal cancer cells [14, 15], which is assumed to be the underlying mechanisms for the antitumor effect of *Dysosma versipellis* extract in our study. This study explored the effect of *Dysosma versipellis* extract podophyllotoxin on the biological behavior of esophageal cancer cells and analyzed its underlying mechanism, aiming to provide experimental evidence for the new drug of esophageal cancer treatment in clinical research.

## 2. Materials and Methods

### 2.1. Experimental Subjects

A total of SPF-graded 30 BALB/C nude mice (Vital River Laboratories, SCXK (Shanghai) 2017–0011), aged 6–8 weeks and weighing 16–19 g, were housed for 7 days with humidity of 60–80% at temperature of 22 ± 2°C, with freedom to eat and drink, in the condition of light exposure and avoidance alternately for 12 h, respectively. All animal experiments were conducted under the approval of Ethics Committee of our hospital and in accordance to the Guide for the Care and Use of Laboratory Animal. Extensive efforts were made to ensure minimal suffering of the animals included in the study. Human esophageal cancer cell CP-C (CP-94251) was purchased from ATCC and the item number was ATCCCRL-4029.

### 2.2. Extraction of *Dysosma versipellis*

The *Dysosma versipellis* (20 kg, No. SJ-JC14619) was purchased from Shanghai Jichun Industrial Co., Ltd. The specific procedures for the extraction method were based on Xu et al. [16], containing extraction, chromatography, and separation. With concentration adjusted to 20 *μ*M, the extract was identified and confirmed as podophyllotoxin by Guangzhou Fuda Detection Center.

### 2.3. Subcutaneous Transplantation Tumor

A total of 30 BALB/C nude mice (class SPF) were equally and randomly divided into the control group, model group, and *Dysosma versipellis* group. CP-C cells (2 × 10^6^ cells in 100 *μ*l) at the concentration of 2 × 10^7^/ml in esophageal cancer were subcutaneously injected into the model group as well as the *Dysosma versipellis* group and same volume of normal saline into the control group. After 7 days, the *Dysosma versipellis* group was intraperitoneally injected with 2 mL *Dysosma versipellis* extract at the concentration of 20 *μ*M once a week. All subjects were treated with *Dysosma versipellis* extract at 8, 15, 22, 29, 36, 43, 50, and 57 days for 8 times and were sacrificed by cervical dislocation after feeding for 60 days. Tumor mass was weighed using an electronic scale (Beijing Jinda Sunshine Technology Co., Ltd.).

### 2.4. Cell Culture Intervention

The esophageal cancer cell medium, composing of 90% high glucose DMEM (containing 4 mM L-glutamine, sodium pyruvate) and 10% fetal bovine serum, was supplied by the North Nano Biological Co., Ltd. and was cultured at 37°C in 95% air and 5% carbon dioxide. CP-C cells in logarithmic growth were selected and divided into 4 groups: control group, podophyllotoxin group, Wnt activator group, and combined group (mixture of podophyllotoxin and Wnt activator). Wnt activator methyl vanillate was purchased from CSNpharm with item number CSN23594 and concentration of 5 mL.

### 2.5. In Vitro Cell Viability Experiment Using MTT

Esophageal cancer cells were made into 4 × 10^6^ cells/mL cell suspension with one for each array and routinely inoculated. The cells were treated with varying concentrations of podophyllotoxin (0.01, 0.1, 0.2, 0.4, and 0.8 *μ*M) for 48 h to evaluate the IC50 of podophyllotoxin at 48 h. The constituent of samples were as follows. Control group: 200 *μ*L cell suspension; podophyllotoxin group: 20 *µ*L podophyllotoxin at the concentration of 0.2 *μ*M + 180 *µ*L cell suspension; Wnt activator group: 20 *μ*L methyl vanillate + 180 *μ*L cell suspension; combined group: 10 *μ*L podophyllotoxin at the concentration of 0.2 *μ*M + 10 *μ*L methyl vanillate + 180 *μ*L cell suspension. Samples in each group were cultured in the 96-well plate for 12 h, 24 h, 48 h, and 72 h, respectively; then, 20 *μ*L MTT (5 mg/mL) solution was added to remove the supernatant containing impurities, dimethyl sulfoxide solution was filled into samples and placed on a horizontal shaking table for 10 min, and then, absorbance at a wavelength of 570 nm was measured by a microplate reader (Shanghai Spark Biotechnology Co., Ltd.). MTT assay kit was purchased from Beijing Equation Jiahong Technology Co., Ltd.

### 2.6. Cell Apoptosis Experiment Using Flow Cytometry

Esophageal cancer cells were digested with 0.25% trypsin and washed twice with PBS, and 100 *μ*L binding buffer was added to prepare a suspension of 1 × 10^6^ cells/mL, followed by addition of 5 *μ*l Annexin V and 5 *μ*l propidium iodide (PI) (Shanghai Yisheng Biotechnology Co., Ltd., 40302ES20). Then, samples were incubated at room temperature for 5 min in the dark and detected using the FC500MCL flow cytometry system (FACS Canto II, USA). Independent experiment of each sample was repeated 3 times to take the average.

### 2.7. In Vitro Cell Invasion Experiment Using Transwell Assays

Cell suspension (5 × 10^5^/mL) was prepared with 100 *μ*L cells seeded into the chamber of transwell coated with Matrigel, and the number of cell-penetrating was calculated after 24 hours, and 3 independent experiments were performed simultaneously. Transwell chamber was purchased from Shanghai Shengbo Biomedical Technology Co., Ltd.

### 2.8. Western Blot

The protein in tissues or cells was extracted by the repeated freeze-thaw method, and protein concentration was determined via the BCA method. With protein concentration adjusted to 4 *μ*g/*μ*L, proteins were separated by 12% polyacrylamide gel electrophoresis with initial voltage of 90 V; then, samples were moved to the appropriate position of the separation gel with voltage elevated to 120 V. After electrophoresis, film formation was performed under the constant pressure of 100 V for 100 min and blocked at 37°C for 60 min. Then, the transfer membrane was sealed off for 2 h using 5% skim milk powder. With immune reaction carried out, the membrane reacted with primary antibody (1 : 1000), incubated at 4°C overnight, washed three times with PBS buffer for 5 min each time the next day, and then incubated with the secondary antibody (1 : 1000) at room temperature for 1 h. Final developing and fixing were carried out using ECL luminescent reagent. Gray value of each band was quantified and analyzed using Quantity One software. Relative expression level of the protein was calculated by the target band gray value/band gray value of internal reference. BCA protein kit, ECL luminescence kit, and trypsin were purchased from Thermo Scientific™, with product numbers 23250, 35055, and 90058, respectively. The primary antibodies including rabbit anti-Wnt, anti-*β*-catenin, anti-GSK3*β*, anti-p-GSK3*β*, and *ß*-actin were purchased from Abcam, Cambridge, UK, with Catalog items ab219412, ab32572, ab75814, ab32391, and ab8226, respectively. The goat anti-rabbit IgG (ab6721, Abcam) was selected as secondary antibody.

### 2.9. Statistical Approach

All statistical analyses in this research were performed using the SPSS19.0 (Asia Analytics Formerly SPSS China), in which measurement data were presented in terms of (mean ± standard deviation). Student's *t*-test was applied in group comparison. ANOVA for repeated measures was employed in the comparison within groups at different time points. Single factor variance was applied in multigroup comparison, and LSD was used in the post hoc test. *P* < 0.05 was considered as statistical significance.

## 3. Results

### 3.1. *Dysosma versipellis* Extracts Attenuate Subcutaneous Tumorigenesis of Esophageal Cancer in Mice

The tumorigenesis rates of the control group, model group, and *Dysosma versipellis* group were 0%, 90% (1 tumor-free mouse), and 80% (2 tumor-free mice), respectively. The tumor mass in the model group (*n* = 9) and *Dysosma versipellis* group (*n* = 8) was (0.38 ± 0.02) g and (0.20 ± 0.02) g, respectively. The tumor mass in the *Dysosma versipellis* group was significantly less than that in the model group (*P* < 0.05, Figures 1(a)–1(c)).

### 3.2. Activation of the Wnt Signaling Pathway in Mice with Subcutaneous Tumorigenesis of Esophageal Cancer Cells

According to the results of Western blot, the expression level of Wnt in the tumor tissue of the model group (*n* = 9) was higher than that in the *Dysosma versipellis* group (*n* = 8). The expression level of *ß*-catenin in tumor tissue of the model group (*n* = 9) and *Dysosma versipellis* group (*n* = 8) was (0.870 ± 0.012) and (0.701 ± 0.017), respectively. Compared to the *Dysosma versipellis* group (*n* = 8), the higher expression level of p-GSK3*β*/GSK3*β* was revealed in the model group (*n* = 9). Expression level of Wnt, *ß*-catenin, and p-GSK3*β*/GSK3*β* in tumor tissue of the *Dysosma versipellis* group was lower than that in the control group (*P* < 0.05, Figure 2).

### 3.3. *Dysosma versipellis* Extracts Inhibit Esophageal Cancer Cell Viability

According to MTT assays, cell viability was decreased as the concentration of podophyllotoxin was increased (Figure 3(a)), and IC 50 of podophyllotoxin in esophageal cancer cells was 0.2 *μ*M, which was used in subsequent experiment in our study. Significant differences in cell viability exhibited among four groups. The viability of esophageal cancer cell in the Wnt activator group was the highest one. The podophyllotoxin group revealed the lowest viability at all-time points compared to the other three groups (*P* < 0.05, Figure 3(b)), suggesting podophyllotoxin can effectively inhibit, while Wnt activators can effectively promote the viability of esophageal cancer cells.

### 3.4. *Dysosma versipellis* Extracts Induce Esophageal Cancer Cell Apoptosis

According to in vitro apoptosis assays, significant differences in cell apoptosis exhibited among four groups. Cell apoptosis rate in the Wnt activator group, control group, and combined group was lower than that in the podophyllotoxin group (*P* < 0.05, Figure 4). In addition, the Wnt activator group indicated the lowest cell apoptosis rate. The data suggested that podophyllotoxin can effectively promote while Wnt activators can effectively inhibit apoptosis of esophageal cancer cells.

### 3.5. *Dysosma versipellis* Extracts Inhibit Esophageal Cancer Cell Invasion

According to in vitro invasion assays, significant differences in the numbers of transmembrane cell exhibited among four groups. It was found that the podophyllotoxin group showed lower numbers of transmembrane cell compared to the remaining three groups (*P* < 0.05, Figure 5) The Wnt activator group showed the highest level. These findings indicated that podophyllotoxin can effectively inhibit, while Wnt activators can effectively promote invasion of esophageal cancer cells.

### 3.6. *Dysosma versipellis* Extracts Inhibit the Activation of the Wnt Signaling Pathway in Esophageal Cancer

According to results of Western blot, significant differences in the expression level of Wnt, *ß*-catenin, and p-GSK3*β*/GSK3*β* exhibited among four groups. The Wnt, *ß*-catenin, and p-GSK3*β*/GSK3*β* expression in the combined group, blank group, and Wnt activator group showed a higher level than the podophyllotoxin group (*P* < 0.05, Figure 6). Podophyllotoxin can effectively inhibit activation of the Wnt signaling pathway.

## 4. Discussion

Recent years, plant active ingredients with little toxicity in Chinese herbal medicines, which is frequently used for clinical treatment due to its ability to inhibit growth and proliferation of cancer cells, have drawn great attention among public [17, 18]. *Dysosma versipellis* is a unique podophyllum plant of barberry family in China, which features excellent biological activity and serves as a new anticancer drug [19]. Yet, few reports have been conducted on its function in malignant tumor, let alone esophageal cancer. Given *Dysosma versipellis* is a valuable and rare species in China, identifying its active ingredients is of a great significance for the rational application. Podophyllotoxin is an active constituent in *Dysosma versipellis*. Xu et al. [16] extracted 15 active constituents of *Dysosma versipellis* and determined that podophyllotoxin has the strongest antiproliferative effect and is capable of inducing tumor cell apoptosis in prostate cancer, breast cancer, gastric cancer, as well as fibroblasts in mouse embryo. In this study, we extracted podophyllotoxin in *Dysosma versipellis* according to the method of Xu and investigated its effect on the growth of esophageal cancer using subcutaneous transplantation experiment. The result showed that the growth rate of subcutaneous esophageal cancer tumors in mice significantly inhibited after the intervention of podophyllotoxin, suggesting antitumor activity of podophyllotoxin in esophageal cancer. We further analyzed the effect of podophyllotoxin on biological behavior of esophageal cancer cells and discovered that podophyllotoxin can inhibit cell viability and invasion, which promotes apoptosis of esophageal cancer cells. Guerram et al. [20] also documented that deoxydipurine has strong in vitro cytotoxic activity and is able to exert the antiglioma effect by inducing cell cycle arrest and apoptosis in G2/M. Taken together, it is basically recognized that *Dysosma versipellis* extract, podophyllotoxin, has an excellent antitumor effect.

At present, there are few reports on the antitumor mechanism of podophyllotoxin, while the Wnt signaling pathway has been reported to be closely associated with the development of esophageal cancer in many studies. Cao et al. [21] reported that naked cuticle homolog 2 can inhibit the proliferation, colony formation, cell invasion and migration, as well as induce G1/S point arrest of esophageal cancer cells by inhibiting the activation of the Wnt signaling pathway. Zhang et al. [22] also confirmed that DACT 2 can inhibit the growth of esophageal cancer via the Wnt signaling pathway. As a result, we hypothesized that regulation of the Wnt signaling pathway is also a mechanism of podophyllotoxin against esophageal cancer. According to the result of several experiments, compared with the intervention of podophyllotoxin alone, the joint use of podophyllotoxin and Wnt signaling activator could restore cell proliferation and invasion ability to some extent and significantly reduce the level of apoptosis in esophageal cancer. However, compared with esophageal cancer cells without any intervention, the viability and invasion ability of esophageal cancer cells in the combined group were inhibited and levels of apoptosis were increased, suggesting that Wnt signaling activators can antagonize the cytotoxicity of podophyllotoxin, and inhibiting the Wnt signaling pathway is one of the mechanisms by which podophyllotoxin exerts cytotoxicity. However, there are no similar reports at present. We expect more similar studies in the future to verify our result. Furthermore, another mechanism of *Dysosma versipellis* extract was investigated in the study of scholar Liang [23], in which researchers extracted kaempferol from *Dysosma versipellis* and determined that kaempferol could inhibit angiogenesis by suppressing expression of vascular endothelial growth factor receptor 2 in human umbilical vein endothelial cells. It is well known that inhibition of angiogenesis plays an extremely important role in treating tumors given it is able to block the blood supply of tumor tissues, thereby “starving” the tumor cells to “death” [24, 25]. We would like to see the same effect of podophyllotoxin be determined in future studies.

However, there still exist some limitations in this study. We only verified the therapeutic effect of *Dysosma versipellis* extracts on esophageal cancer in the cell and animal model, and further clinical validation remains to be investigated. Besides, investigation of Wnt activator resisting to antitumor effects of *Dysosma versipellis* extracts on esophageal cancer should be considered gravely in further study, since we proposed the antitumor effects of *Dysosma versipellis* extracts achieved by regulating the Wnt signaling pathway. Moreover, in vitro experiments based on multiple types of esophageal cancer cells should be performed further to avoid single-cell bias during result interpretation. In summary, podophyllotoxin in *Dysosma versipellis* has an excellent antiesophageal cancer effect. It is able to inhibit cell viability and invasion to promote apoptosis of esophageal cancer cells by inhibiting the Wnt signaling pathway, which could be potentially used in future clinical treatment of esophageal cancer.

## Figures and Tables

**Figure 1:** *Dysosma versipellis* extracts attenuate subcutaneous tumorigenesis of esophageal cancer in mice. ∗*P* < 0.05.

**Figure 2:** *Dysosma versipellis* extracts inhibit the activation of the Wnt signaling pathway in mice subcutaneous tumorigenesis of esophageal cancer. ^∗^*P* < 0.05 compared with the control group and ^#^*P* < 0.05 compared with the model group.

**Figure 3:** *Dysosma versipellis* extracts inhibit esophageal cancer cell viability. ^∗^*P* < 0.05.

**Figure 4:** *Dysosma versipellis* extracts induce esophageal cancer cell apoptosis. ∗, #, and & refer to *P* < 0.05 compared with the blank group, podophyllotoxin group, and Wnt activator group, respectively.

**Figure 5:** *Dysosma versipellis* extracts inhibit esophageal cancer cell invasion. ∗, #, and & refer to *P* < 0.05 compared with the blank group, podophyllotoxin group, and Wnt activator group, respectively.

**Figure 6:** *Dysosma versipellis* extracts inhibit the activation of the Wnt signaling pathway in esophageal cancer cells. ∗, #, and & refer to *P* < 0.05 compared with the blank group, podophyllotoxin group, and Wnt activator group, respectively.

## Data Availability

The data used to support the findings of this study are included within the article.
